The article "Recent Evidence of Tea Tree Oil Effectiveness in Blepharitis Treatment" was published in 2022. Journal: Biomed Res Int.

# Recent Evidence of Tea Tree Oil Effectiveness in Blepharitis Treatment

**DOI:** 10.1155/2022/9204251

**Published:** 2022-07-30

**Authors:** Luigi Capasso, Giulia Abbinante, Alessia Coppola, Giulio Salerno, Maddalena De Bernardo

**Affiliations:** ^1^UOC Oculistica, Ospedale del Mare ASL Napoli 1 Centro, Napoli, Italy; ^2^Department of Medicine, Surgery and Dentistry, “Scuola Medica Salernitana”, University of Salerno, Baronissi, SA, Italy

## Abstract

The purpose of our study is to see how beneficial is tea tree oil (TTO) for treating chronic blepharitis topically, with a focus on the Demodex mite. To discover all possibly relevant published papers, an accurate Pubmed database search analysis of the current literature was undertaken from 2012 to December 2021. Fourteen papers dealing with the use of TTO to treat chronic blepharitis have been found. The effectiveness of TTO treatment was tested in vitro by 4 authors and in vivo by 10 authors. All studied confirmed efficacy of TTO treatment, even cyclic, on Demodex mite blepharitis. TTO can be used for lid scrubs, facial cleanser, eyelid patch, eyelid gel, eyelash shampoo or, more commonly, as TTO impregnated eyelid wipes. The scientific evidence of TTO for chronic blepharitis treatment gives a lot of confidence for the progress that this treatment may have in the future clinical practice.

## 1. Introduction

Itching, flaking, redness, burning, and crusting of the eyelids are major symptoms of blepharitis, a common inflammatory illness of the eyelid edge, with a chronic course.

Chronic blepharitis is usually divided into two types: anterior blepharitis, which affects the anterior lid edge and eyelashes, and posterior blepharitis, which affects the meibomian gland. [1]

The Demodex mite is a commensal organism of the skin bacterial flora, which does not give symptoms in normal conditions, but in some eyelid tissues, its presence may cause inflammatory process [2].

Demodex's pathogenetic implication in the blepharitis inflammatory process is explored [3]. The life cycle from egg to adult mite lasts between 14 and 18 days. The eggs are laid in the sebaceous glands and hair follicles and then turn into larvae until they reach the adult form. When demodicosis sets in, the primary symptom is eyelid itching, which may be accompanied by blepharitis, eyelid swelling, and eye discomfort [4]. Demodex is divided into two species that produce anterior and posterior blepharitis, respectively: *Demodex follicolorum* and *Demodex brevis*. *D. follicolorum* reproduces around the hair follicles, instead *D. brevis* reproduces around the sebaceous glands [5].

Tea tree oil (TTO) is a fragrant essential oil derived from the leaves of Melaleuca alternifolia, a Myrtaceae plant.

The article "Recent Evidence of Tea Tree Oil Effectiveness in Blepharitis Treatment" was published in 2022. Journal: Biomed Res Int.

The main constituent of TTO is represented by terpinen-4-ol (T4O), present in concentrations ranging from 30% to 48%. This component is the most active in killing Demodex mites, including larvae and eggs. It also possesses antibacterial, antifungal, anti-inflammatory, and acaricidal activity [6, 7].

To be able to cure blepharitis before anterior segment ocular surgery, such as cataract extraction [8, 9] or refractive surgery [10–13], could be very important [14, 15], primarily to lower the chance of endophthalmitis.

In fact, microorganisms of the eyelid edge, conjunctiva, and tear film, particularly gram-positive bacteria, predominantly coagulase-negative Staphylococcus spp., are the most common cause of acute postoperative endophthalmitis [16].

As a result, in addition to preoperative topical antibiotics and antiseptic povidone–iodine (PVI) 5% topically applied to the cornea and conjunctival sac, eyelid disinfection can be utilized as an additional prophylactic method to avoid ocular infections [17].

In the case of such a situation, the effect of TTO-based drugs has been recorded in various articles. The purpose of this study was to assess the efficacy of TTO in the chronic blepharitis topical therapy, with a focus on the Demodex mite.

## 2. Materials and Methods

To find all potentially relevant published papers, a Pubmed database literature search was conducted from 2012 to December 2021. The following keywords were utilized in the search approach: blepharitis, lid, tea tree oil, and TTO. Additional pertinent papers were found by scanning the references cited in the recovered articles.

## 3. Results and Discussion

From this search, 14 papers dealing with the use of TTO to treat chronic blepharitis have been found.

### 3.1. Studies In Vitro

The effectiveness of TTO treatment was tested in vitro by four authors [18–21], and it is summarized in Table 1.

Cheung et al. [18] conducted a randomized in vitro investigation on 93 live Demodex mites extracted from the lashes of ten previously epilated volunteers. After applying four eyelid detergents (Cliradex® towelette cleanser, OustTM Demodex® cleanser, BlephadexTM eyelid foam, and TheraTears® SteriLid® eyelid cleanser) and four antimicrobial solutions, the mites' vitality was evaluated for 300 minutes based on limb and body movement and crenated or translucent appearance (100% undiluted and 50% diluted Home Essentials TTO, 100% T4O, and 100% linalool). The 50% diluted TTO solution was made by combining undiluted TTO and Healtheries Almond Oil in a 1 : 1 ratio. As a negative control, untreated mites were tested.

Cheung then used Kaplan-Meier survival assessment and mass spectrometry analysis to measure the anti-Demodex chemicals' absolute and relative concentrations, as well as the T4O content of commercial detergents and TTO. As a result, no significant changes in undiluted TTO, T4O, or linalool were found (all *p* > 0.05).

The article "Recent Evidence of Tea Tree Oil Effectiveness in Blepharitis Treatment" was published in 2022. Journal: Biomed Res Int.

T4O and undiluted linalool demonstrated similar antiparasitic effectiveness. Even though all commercial eyelid cleansers reduced mite survival rates compared to the untreated group, Cliradex showed the strongest antidemodectic action in vitro and the highest T4O level of the four eyelid cleansers, whereas linalool was only found in TheraTears® SteriLid®.

Chen et al. [19] studied in vitro the potential toxicity of T4O on epithelial cells of the meibomian glands, cultured with variable concentrations (1.0%, 0.1%, and 0.01%) of T4O under conditions of proliferation or differentiation up to 5 days, with analysis of cellular presence, persistence, P-Akt signaling, accumulation of lysosomes, and content of neutral lipids. This resulted in significant in vitro toxicity for all concentrations tested. This result confirms the authors' initial hypothesis, namely, that the toxicity of TTO on nonocular epithelial cells can also extend to the epithelial cells of the meibomian glands.

Su et al. [20] evaluated the antibacterial effectiveness of a 2 percent T4O formulation against pathogens mentioned in Chapter 51 of the United States Pharmacopeia (USP <51>) by Alcami Corporation in vitro (Wilmington, North Carolina, USA). The log 2.0 decrease rate was used to assess microorganism decrease at days 14 and 28. They also studied cutaneous and ocular irritation using the repeated insult patch test (RIPT) with 2 percent T40 and the Hen's Egg chorioallantoic membrane test, respectively. The dermal reactions of the RIPT were recorded based on a 6-point scale that evaluated absence (0 points) or the presence of a mild, moderate, marked, or severe skin reaction. No sign of irritation, allergy, or any other cutaneous response was detected or described by any of the 55 participants after exposure to 2% T4O, whereas only three of the 58 subjects stopped for personal reasons. In the second test, ocular irritation was measured using two scores: an irritation score based on the time of appearance of the adverse reactions (hemorrhage, vascular lysis, and coagulation) and a severity score based on the severity of adverse reactions after 1 and 5 minutes. The HET-CAM test was used to assess ocular irritation, and the results revealed that the T4O 2% formulation was both safe and effective at destroying pathogens related to eye disorders.

More recently, Bulut and Tanriverdi [21] examined the in vitro properties of tea tree oil active components in eye washing wipes and solutions on Demodex life span. The concentrations of terpinem-4-ol (T40), 2.5%TTO, and 7.5% TTO in the examined preparations were 0.5%, 2.5%, and 7.5%, respectively. They found that T4O had an adequate anti-Demodex action even at extremely low dilutions (0.5%).

The article "Recent Evidence of Tea Tree Oil Effectiveness in Blepharitis Treatment" was published in 2022. Journal: Biomed Res Int.

The antiparasitic action of TTO against ocular Demodex is confirmed in all in vitro investigations, but they have significant limitations because the clinical effectiveness of TTO in treating eye disorders has not been directly explored, and the preparation has not been tested right on eyelid skin and margin. Even though a lower concentration of T4O is improbable to induce skin or ocular irritation, clinical trials to assess the advantages and risks of daily usage of T4O on the eyelid margins are needed, according to Chen et al.

### 3.2. Studies In Vivo

The effectiveness of TTO treatment was then also tested in vivo by several authors [22–31] and reviewed in Table 2.

In a case-control study, Maher [22] assessed the efficacy of lid washing with a TTO compound (Naviblef) in 40 subjects with blepharitis and meibomian gland dysfunction. The patients were split into two groups, each with 20 patients. One group received Naviblef treatment, while the other received merely eye massage and washing. The signs and symptoms of all patients treated with TTO mixture lid cleaning significantly improved, as well as tear film stability (*p* < 0.001). On the contrary, only five patients showed improvement in the other group, without statistically significant changes.

In 135 patients with Demodex mite blepharitis, Karakurt and Zeytun [23] investigated the effectiveness of a 7.5 percent TTO eyelash wash. Eyelash shampoo was used on all the patients, some with TTO and some without this oil. Those treated with TTO showed a statistically significant reduction (*p* < 0.001) in Demodex mite by 36%, with an average count reduced from 6.33/cilia to 0. In those not treated with TTO, however, the mean decreased from 12.46/lash to 4.15/lash (*p* < 0.001). Finally, TTO eyelash shampoo was found to be three times more active in reaching total Demodex reduction, particularly in terms of Demodex count and ocular discomfort.

Ergun et al. [24] investigated the efficacy of two TTO-based washing ointments in 49 patients with chronic blepharitis who were separated into two groups. Group 1 (25 subjects) received a base gel with 3% (*w*/*w*)-TTO, while group 2 (24 participants) received an enhanced gel with 3% (*w*/*w*)-TTO plus essential oils and vitamins. The authors measured the ocular surface disease index (OSDI), tear breaking time (TBUT), ocular surface staining pattern, Schirmer's test, impression cytology, Demodex presence, and TNF-, IL-6, and IL-1 levels at the initial visit and after one month of treatment. There was an improvement in all parameters, with greater reduction of cytokines and Demodex counts in group 2.

The article "Recent Evidence of Tea Tree Oil Effectiveness in Blepharitis Treatment" was published in 2022. Journal: Biomed Res Int.

Koo et al. [25] studied 335 patients with ocular discomfort by evaluating their OSDI score and found Demodex blepharitis in 84% of patients with ocular symptoms. Eyelid lavage with TTO (106 patients) or without TTO (control group, 54 patients) was given to the latter for a month in random fashion. Patients treated with TTO showed a significant reduction in Demodex count and improvement in ocular symptoms. The control group also showed a decrease in Demodex count after treatment, but it was less reduced than the TTO group.

Alver et al. [26] used 39 chronic, treatment-refractory Demodex blepharitis patients who were treated with 4% TTO eyelid gel and 10% eyelash shampoo to try to develop a systematic grading method for a very precise diagnosis of Demodex blepharitis. Demodex follicolorum was detected in 30 patients by light microscopy. The authors created a table in which they entered the symptoms (burning, sting, itching, and pain), the localization of blepharitis (anterior or posterior), and additional points (evaluation of eyelashes, ocular surface, and cornea). TBUT, OSDI, keratitis, epithelial defects, and blepharitis were evaluated at the time of diagnosis and after one month. TTO therapy resulted in resolution of symptoms in 25 patients, and treatment was recommended for all those with a score >4, based on the table devised by the authors.

Murphy et al. [27] evaluated 86 patients, divided into three groups to compare the efficacy of the Dr Organic Tea Tree facial cleanser, OcuSoft Lids Scrub Plus, and the BlephEx TM device in the treatment of follicular blepharitis by Demodex. Patients were assessed after two and four weeks of treatment. Ocular symptoms were clearly reduced in all three groups during the second week of treatment and continued to diminish after four weeks of treatment. There was a significant decrease of Demodex levels in all three groups at the end of treatment.

Mergen et al. [28] compared tea tree oil and chamomile oil swabs to baby shampoo (BS) in patients with seborrheic blepharitis in a double-blind randomized clinical experiment. For 8 weeks, 23 patients were given BS, and 26 were given swabs, followed by 4 weeks of therapy discontinuation. For the treatment of seborrheic blepharitis, both groups of patients exhibited equivalent efficacy.

Concerning Demodex and symptoms decrease, swabs showed better results. It is worth noting that skipping four weeks of therapy may not result in a recurrence of symptoms or Demodex infestation.

The article "Recent Evidence of Tea Tree Oil Effectiveness in Blepharitis Treatment" was published in 2022. Journal: Biomed Res Int.

In a prospective study, Liu and Gong [29] compared the antidemodectic benefits of okra eyelid patch with tea tree oil in Demodex blepharitis (TTO). An okra eyelid patch (27patients) or an eye care patch soaked with terpinen-4-ol (T4O), the major element of TTO (25 controls) were given to 52 Demodex blepharitis patients with ocular discomfort for three months. Despite the fact that the two therapies are identical, the authors claim that the okra eyelid patch may be better for sensitive Demodex blepharitis patients, such as the elderly and children.

On Demodex blepharitis, Evren Kemer et al. [30] explain the success of cyclic therapy of heat followed by terpinen-4-ol soaked wipes to eyelids (twice a day for 2 weeks, then the same treatment was repeated after a 7–10 day break). The identical procedure was followed once more. After the first and second therapy cycles, as well as after a year, the patients were assessed. After the first cycle of treatment, tear breakup time, Schirmer, lid margin score, ocular surface disease index, Oxford grade, and meibomian gland expressibility scores all improved statistically significantly (*p* < 0.05). The patients' symptoms and tear function tests improved dramatically following the second cycle compared to pretreatment levels. Symptoms returned in two patients (93%) after a 12-month follow-up.

In fifty patients with Demodex blepharitis, Jacobi et al. [31] evaluated a combined treatment utilizing eyelid wipes impregnated with 2.5% terpinen-4-ol (T4O) and 0.2% hyaluronic acid (HA) for 28 days, investigating the continuation of the treatment effect utilizing of eyelid cleansing wipes. They found that daily treatment with T4O impregnated eyelid wipes relieved ocular symptoms and signs lowering the mite count in individuals with Demodex blepharitis after four weeks. Following that, a 4-week maintenance treatment with wipes sustained or enhanced the treatment's success.

All studies confirmed that patients with Demodex blepharitis treated by different formulation of TTO (eyelash shampoo, eyelid wipes, and eyelid patch) had a significant reduction in Demodex count and an improvement in ocular signs and symptoms, concluding that this therapy is both safe and effective in medical settings.

## 4. Conclusions

There is a lot of interest these days in producing natural medicinal solutions with small adverse effects. The scientific evidence of TTO for chronic blepharitis treatment and the interest of pharmaceutical companies to conceive new formulation of this essential oil give a lot of confidence for the progress that this treatment may have in the future clinical practice.

The article "Recent Evidence of Tea Tree Oil Effectiveness in Blepharitis Treatment" was published in 2022. Journal: Biomed Res Int.

## Figures and Tables

**Table 1:** Summary chart of effectiveness of TTO treatment tested in vitro.

Author	Purpose of study	Results
Cheng et al.	To assess the vitality of 93 live Demodex mites for 300 minutes, based on limb and body movement and crenated or translucent appearance, after the application of four eyelid cleansers and four antimicrobial solutions (TTO 50% diluted and 100% undiluted, T4O, linalool).	No significant differences were observed between undiluted TTO, T4O, and linalool (*p* > 0.05) undiluted linalool and T4O showed comparable antiparasitic efficacy.
Chen et al.	To evaluate the potential toxicity of T4O on epithelial cells of the meibomian glands with variable T4O concentrations (1.0%, 0.1%, and 0.01%).	TTO is toxic on nonocular epithelial cells and on epithelial cells of the meibomian glands for all tested concentrations.
Su et al.	Alcami corporation wanted to evaluate the antibacterial activity of a 2% T4O formulation against pathogens specified in chapter 51 of the United States Pharmacopeia (USP 51>).	T40 2% formulation is safe and effective in rapidly killing microorganisms associated with ocular diseases.
Bulut and Tanriverdi	The purpose of this study was to see how TTO active components in eye washing wipes and mixtures affected Demodex life span.	Even at relatively low doses, T4O has an anti-Demodex action (0.5%).

**Table 2:** Summary chart of effectiveness of TTO treatment tested in vivo.

Author	Purpose of study	Results
Maher et al.	The effectiveness of lid scrubbing with a TTO solution (Naviblef) was evaluated in 40 patients divided into two groups of 20 patients each, one with blepharitis and meibomian gland dysfunction and the other with healthy subjects in a case-control study.	All patients who received lid scrubbing with a TTO formula had statistically significant improvement in signs and symptoms (*p* > 0.001), while 5 patients only treated with eye massage and cleansing changes had not statistically significant changes (*p* < 0.001).
Karakurt et al.	In 135 individuals with Demodex mite blepharitis, the efficacy of a 7.5% TTO eyelash wash was investigated.	TTO eyelash shampoo was found to be three times more efficient in reaching total Demodex elimination, lowering Demodex count and ocular symptoms dramatically.
Ergun	To assess the efficacy of two TTO-based cleaning gels in two groups of 49 individuals with chronic blepharitis. Group 1 (50 eyes of 25 patients) received a basic gel with 3% (*w*/*w*)-TTO, whereas group 2 (48 eyes of 24 patients) received an advanced gel with 3% (*w*/*w*)-TTO plus essential oils and vitamins.	The ocular surface disease index (OSDI), tear breaking time (TBUT), ocular surface staining pattern, Schirmer's test, and impression cytology all improved in group 2, as did the cytokines and Demodex numbers.
Koo et al.	To study 335 patients divided in 2 randomized groups with ocular discomfort to receive eyelid lavage with or without TTO, by evaluating the OSDI score	Demodex blepharitis was present in 84% of patients with ocular symptoms. Patients treated with TTO showed a significant reduction in Demodex count and improvement in ocular symptoms, more evident than the other group.
Alver et al.	Enrolling 39 chronic, treatment–refractory Demodex blepharitis patients undergoing therapy with 4% TTO eyelid gel and 10% eyelash shampoo to develop a scoring system for a very precise diagnosis of Demodex blepharitis.	TTO therapy resulted in resolution of symptoms in 25 patients, and treatment was recommended for all those with a score >4, based on the table proposed by the authors.
Murphy et al.	The purpose of this study was to examine the efficacy of the Dr Organic Tea Tree face cleanser, OcuSoft Lids Scrub Plus, and the BlephEx TM device in the treatment of follicular blepharitis in 86 patients divided into three groups. For four weeks, the participants were instructed to wipe their eyes every night.	At the end of therapy, all three groups had considerably lower Demodex numbers.
Mergen et al.	In patients with seborrheic blepharitis, swabs containing tea tree oil and chamomile oil were compared to baby shampoo (BS).	In terms of Demodex reduction and clinical improvement, patients in both groups demonstrated equivalent success in the treatment of seborrheic blepharitis.
Liu and Gong	To compare the antidemodectic benefits of an okra eyelid patch to tea tree oil in a prospective trial of Demodex blepharitis.	Sensitive Demodex blepharitis patients, such as the elderly and children, may benefit from the use of an okra eyelid patch.
Evren Kemer et al.	On Demodex blepharitis, the effectiveness of cyclic therapy of heat followed by terpinen-4-ol soaked wipes to eyelids (twice a day for 2 weeks, then 7-10 days off, then the same treatment was repeated) was investigated.	The patients' symptoms and tear function tests improved dramatically following the second cycle compared to premedication stages. Symptoms recurred in two subjects (93%) after a 12-month follow-up.
Jacobi et al.	In fifty patients with Demodex blepharitis, the management of eyelid wipes filled with 2.5% terpinen-4-ol (T4O) and 0.2% hyaluronic acid (HA) for 28 days was evaluated.	During the initial treatment phase, daily use of T4O filled eyelid wipes considerably relieved ocular symptoms and signs, while also lowering the mite count.
